The article "Establishment and Analysis of a Prognostic Model of Autophagy-Related lncRNAs in ESCA" was published in 2022. Journal: Biomed Res Int.

# Establishment and Analysis of a Prognostic Model of Autophagy-Related lncRNAs in ESCA

**DOI:** 10.1155/2022/9265088

**Published:** 2022-07-26

**Authors:** Feifei Chen, Jian Zhang, Wenxia Bai

**Affiliations:** ^1^Department of Gastroenterology, The Affiliated Jiangning Hospital of Nanjing Medical University, Nanjing 211100, Jiangsu, China; ^2^Department of Echocardiography, Zhongshan Hospital, Fudan University, Shanghai Institute of Cardiovascular Diseases, Shanghai Institute of Medical Imaging, Shanghai 200000, China

## Abstract

Esophageal cancer (ESCA) is a malignant tumor of the upper gastrointestinal tract, with a high mortality rate and poor prognosis. Long noncoding RNAs (lncRNAs) play a role in the malignant progression of tumors by regulating autophagy. This study is aimed at establishing a prognostic model of autophagy-related lncRNAs in ESCA and provide a theoretical basis to determine potential therapeutic targets for ESCA. The transcriptome expression profiles were downloaded from The Cancer Genome Atlas (TCGA). We identified autophagy-related mRNAs and lncRNAs in ESCA using differential expression analysis and the Human Autophagy Database (HADb). Four differentially expressed autophagy-related lncRNAs with a prognostic value were identified using Cox regression and survival analyses. Furthermore, the combination of the selected lncRNAs was able to predict the prognosis of patients with ESCA more accurately than any of the four lncRNAs individually. Finally, we constructed a coexpression network of autophagy-related mRNAs and lncRNAs. This study showed that autophagy-related lncRNAs play an important role in the occurrence and development of ESCA and could become a new target for the diagnosis and treatment of this disease.

## 1. Introduction

Esophageal cancer (ESCA) is an aggressive malignant gastrointestinal tumor that affects the epithelial tissue of the esophagus [1], with a high mortality rate and poor prognosis, causing more than 500,000 deaths annually [2]. At present, the diagnosis of ESCA relies mainly on gastroscopy and pathological evidence. However, ESCA symptoms are often discrete in the early stages of the disease and are mostly diagnosed during the late and advanced stages. Despite treatments such as surgery and neoadjuvant chemotherapy, the survival rate of ESCA remains low [2]. Therefore, it is important to understand the mechanism underlying the occurrence and development of ESCA and identify biomarkers for its diagnosis and prognosis.

Autophagy is a survival-promoting pathway that functions in the capture, degradation, and circulation of intracellular proteins and organelles in the lysosomes [3]. Autophagy retains the functions of organelles, prevents the toxic accumulation of cellular waste products, and provides a substrate for maintaining metabolism during starvation [4]. The role of autophagy in cancer depends on the availability of nutrients, microenvironmental pressure, and the immune system. Although autophagy inhibits tumorigenesis in some cancers, it promotes this process in most cancers [5, 6]. Wu et al. demonstrated that the tight junction protein CLDN1 activates AMPK/STAT1/ULK1 signaling in the esophageal squamous cell carcinoma cell lines TE10 and TE11, which induces autophagy in esophageal squamous cell carcinoma cells, and enhances cancer cell proliferation and metastasis [7]. Several studies reported that autophagy is upregulated in hypoxic tumor areas, inhibits tumor-induced inflammation, promotes tumor cell survival, and increases growth and invasiveness [8, 9]. Another study reported altered expression of autophagy markers in patients with ESCA and a significant association between microtubule-associated light chain 3 (LC3), the most characteristic autophagy marker in ESCA, and poor survival in these patients [10]. Therefore, autophagy-related genes are potential targets for the treatment of ESCA and have broad prospects for clinical applications.

The article "Establishment and Analysis of a Prognostic Model of Autophagy-Related lncRNAs in ESCA" was published in 2022. Journal: Biomed Res Int.

At present, the Human Genome Project has deciphered approximately 25,000 genes; however, only approximately 2% of these genes encode proteins, and many are noncoding genes that are transcribed to noncoding RNAs. Among these, those with a sequence length of >200 bp are called long noncoding RNAs (lncRNAs) [11]. Although these genes are not translated into proteins, they play crucial biological roles, such as regulating gene transcription, translation, and shearing processes and regulating microRNA and protein folding [12]. lncRNAs promote the occurrence and development of tumors by regulating tumor cell proliferation, migration, and invasion, modulating the cell cycle, and inhibiting apoptosis [13]. H19 is a classic cancer-promoting lncRNA that mediates the metastasis of ESCA in vitro and in vivo through the STAT3/EZH2/*β*-catenin axis. It is negatively regulated by let-7 at the posttranscriptional level, and its downregulation inhibits the proliferation, migration, and invasion of ESCA cells and promotes apoptosis [14]. UCA1 is another lncRNA that is overexpressed in gastrointestinal cancers and has an important regulatory role in cancer progression by acting as a competing endogenous RNA to regulate the expression of the target protein SOX4, thereby promoting ESCA cell proliferation [15]. UCA1 can also promote the glycolytic process in ESCA cells by sequestering miR-203 and alleviating its inhibitory effect on hexokinase 2 (HK2), thereby increasing HK2 levels and promoting the Warburg effect, cell proliferation, and metastasis [16]. Although most lncRNAs have tumor-promoting effects, some are tumor suppressors that inhibit tumor proliferation and migration and promote tumor cell apoptosis through multiple molecular mechanisms [13]. For example, the NEF overexpression reduces the expression of Wnt/*β*-catenin pathway-related proteins in ESCA cells, thereby inhibiting tumor cell proliferation, migration, and invasion [17]. Uc061hsf.1, a lncRNA, is a tumor suppressor gene and a direct transcriptional target of p53 [18]. Additionally, it regulates the expression of the downstream transcription factor FOXA1 and inhibits the proliferation and migration of ESCA cells [18].

The article "Establishment and Analysis of a Prognostic Model of Autophagy-Related lncRNAs in ESCA" was published in 2022. Journal: Biomed Res Int.

Chen et al. reported that autophagy-related lncRNA prognostic markers, such as AL355574.1, are associated with the immune microenvironment and survival outcomes in patients with gastric cancers [19]. Increasing studies have found that lncRNAs affect the malignant progression of tumors by regulating autophagy [20–24]; however, the specific mechanism by which this regulation occurs remains unclear. Therefore, this study used coexpression analysis of autophagy-related mRNAs and lncRNAs in ESCA to identify autophagy-related lncRNAs, establish a prognostic model, and analyze its correlation with the clinical characteristics and survival of patients with ESCA.

## 2. Materials and Methods

### 2.1. Datasets and Sample Extraction

Transcriptome sequencing data and clinical-related data of patients with ESCA were downloaded from the Cancer Gene Atlas database [TCGA, Repository (http://cancer.gov/)]. The information obtained included the age, sex, survival time, survival status, tumor stage, and grade of patients with ESCA and other clinical data, as well as the transcriptome data of the tumors of 160 patients with ESCA and control samples comprising 11 adjacent tissues. The prcomp function of *R* was used to perform a principal component analysis (PCA).

### 2.2. Screening of Autophagy-Related Differentially Expressed Genes

The “limma” *R* package was used to sort and screen out differentially expressed lncRNAs (DElncRNAs) and mRNAs (DEmRNA) in ESCA using the following criteria: |log_2_ FC > 1| and *P* < 0.05. The list of autophagy genes was obtained from the Human Autophagy Database (HADb, http://autophagy.lu/clustering/index.htm). Autophagy-related DEmRNAs were obtained using the intersection of DEmRNAs and autophagy-associated genes listed on the website (http://bioinformatics.psb.ugent.be/webtools/Venn/). The correlation between lncRNAs and autophagy-related DEmRNAs was calculated using Pearson's correlation. lncRNAs with |r| > 0.3 and *P* < 0.001 were considered autophagy-related lncRNAs. The coexpression network was visualized using Cytoscape 3.7.2.

The article "Establishment and Analysis of a Prognostic Model of Autophagy-Related lncRNAs in ESCA" was published in 2022. Journal: Biomed Res Int.

### 2.3. Identification of Prognostic Autophagy-Related lncRNAs

The prognostic value of autophagy-related lncRNAs was calculated using multiple Cox regression with *P* < 0.05. We constructed a risk score based on the linear combination of autophagy-related lncRNA expression levels multiplied by a regression coefficient. Based on this, participants were divided into high-risk and low-risk groups. Differences in survival between the two groups were compared using the log-rank test.

### 2.4. Development of the Prognostic Model

Univariate and multivariate Cox regression analyses were performed to explore the correlation between the autophagy-related lncRNA risk score and the age, sex, tumor grade, and stage of patients with ESCA. A nomogram was used to predict patient survival. The concordance index (C-index), calibration curves, and receiver operating characteristic (ROC) curves were used to determine the accuracy of the model.

### 2.5. Functional Analysis

Gene set enrichment analysis (GSEA) was conducted using the “clusterProfiler” package in *R* to determine the functional enrichment of autophagy-related lncRNAs. The enrichment plot package was used to visualize the results of Gene Ontology (GO) and Kyoto Encyclopedia of Genes and Genomes (KEGG) enrichment analysis. StarBase (https://starbase.sysu.edu.cn/) and miRWalk (http://mirwalk.umm.uni-heidelberg.de/) website were used to predict the possible downstream targets of candidate lncRNAs.

### 2.6. Statistical Analysis

Statistical analyses were conducted using *R* language (version 3.6). Statistical tests were bilateral, and statistical significance was set at *P* < 0.05.

## 3. Results

### 3.1. Construction of a Coexpression Network

We identified 14142 recognizable lncRNAs, eight of which were downregulated and 53 were upregulated in ESCA (Figure 1(a)). Similarly, 638 DEmRNAs, including 472 with high expression and 166 with the low expression, were identified using TCGA dataset (Figure 1(b)). In total, 257 genes were obtained from the HADb, of which five (*PINK1*, *BIRC5*, *ITPR1*, *PRKAB1*, and *GABARAPL1*) were differentially expressed in ESCA simultaneously; therefore, we defined them as autophagy-related DEmRNAs. We used Pearson's correlation analysis to identify DElncRNAs that have a coexpression relationship with autophagy-related DEmRNAs (|r| > 0.3 and *P* < 0.001; Table 1). Finally, we identified five mRNAs (*PINK1*, *BIRC5*, *ITPR1*, *PRKAB1*, and *GABARAPL1*) and 11 lncRNAs (MAFG-DT, AC007637, AC091563, AC004982, FENDRR, AC037198, SNHG1, SEMA3B, ZNF710, and LINC02381) that might regulate autophagy in ESCA (Figures 1(c) and 1(d)).

The article "Establishment and Analysis of a Prognostic Model of Autophagy-Related lncRNAs in ESCA" was published in 2022. Journal: Biomed Res Int.

### 3.2. Identification of a Prognostic Autophagy-Related lncRNA Signature

According to the results of multivariate Cox regression analysis, four autophagy-related lncRNAs (AC092718, SEMA3B-AS1, FENDRR, and LINC02381) had prognostic value for patients with ESCA (*P* < 0.05). Of these, FENDRR, LINC02381, and SEMA3B-AS1 were prognostic risk factors, and AC092718 was a favorable prognostic factor (Figure 2). The four lncRNAs were used to establish an autophagy-related lncRNA signature. To further evaluate the prognostic value of the four-gene combination in patients with ESCA, the patients were divided into high- and low-risk groups according to the median score of the Cox regression model. The patients' risk scores continued to increase from left to right (Figure 3(b)). According to the survival diagram, patients in the high-risk group had shorter survival times and higher mortality rates than those in the low-risk group (Figure 3(c)). Kaplan–Meier survival analysis also confirmed that the survival time of patients in the high-risk group was significantly shorter than that of patients in the low-risk group (*P* < 0.05; Figure 3(a)). The expression of the four genes in the high- and low-risk groups were presented as a heat map in Figure 3(d). These results suggested that the combination of these four genes can be used as a specific prognostic index for patients with ESCA.

### 3.3. Construction of a Coexpression Network

Cytoscape was used to visualize the coexpression network, which included four lncRNAs and four mRNAs associated with autophagy in ESCA (Figure 4(a)). A hazard ratio (HR) > 1 was considered a risk factor, whereas HR < 1 was considered a protective factor. The Sankey diagram confirmed that FENDRR, LINC02381, and SEMA3B-AS1 were risk factors for patients with ESCA, whereas AC092718 was a protective factor (Figure 4(b)).

### 3.4. Clinical Value of the Autophagy-Related lncRNA Signature

The forest plot of the univariate analysis showed that stage, M, N, and risk scores could predict the prognosis of patients with ESCA (Figure 5(a)). Multivariate Cox analysis showed that only the risk score could be used as an independent prognostic factor (Figure 5(b)). However, ROC curve analysis showed that the area under the curve (AUC) values of the risk model, M, and N were 0.834, 0.544, and 0.646, respectively (Figure 5(d)). Therefore, compared to that with TNM staging, the risk model constructed herein was more accurate in predicting patient survival. As indicated in the nomogram, the risk score was the largest contributor to the 3-and 5-year overall survival rates of patients with ESCA (Figure 5(c)). The C-index of the prognostic model was 0.796 (95% CI: 0.739–0.853), and the 5-year survival rate AUC of the risk score was 0.834, indicating its reliable predictive ability (Figure 5(d)). To investigate the differences and similarities among the grouped samples, PCA was performed based on the expression profiles (Figure 6(a)) and autophagy-related lncRNA prognostic signatures (Figure 6(b)). Collectively, our results indicated that the autophagy-related lncRNA signature might be closely related to the progression and prognosis of ESCA.

The article "Establishment and Analysis of a Prognostic Model of Autophagy-Related lncRNAs in ESCA" was published in 2022. Journal: Biomed Res Int.

### 3.5. Functional Analysis

To investigate the biological characteristics of the proposed lncRNAs, we analyzed GO enrichment analysis using GSEA. GO analysis showed that autophagy-related biological processes such as autophagosome assembly and autophagosome organization were significantly enriched in the ESCA group (Figure 7(a)). Subsequently, we identified 585 possible downstream targets of candidate lncRNAs. The KEGG enrichment analysis of target genes showed that autophagy and mitophagy were significantly enriched and identified pathways that also included pathways in cancer, gastric cancer, endocytosis, and p53 signaling pathways (Figure 7(b)).

## 4. Discussion

ESCA is one of the most malignant cancers worldwide, and China has the highest incidence of ESCA in the world [25]. The incidence of ESCA is associated with age, sex, obesity, eating habits, genetic susceptibility, and other risk factors. Its occurrence and development are multifactorial and complex processes [26]. Therefore, it is necessary to identify new biomarkers to improve its prognosis.

Autophagy-related pathological processes are increasingly being recognized as important disease mechanisms for nonmalignant (neurodegeneration and diffuse lung parenchymal disease) and malignant diseases [27]. Although autophagy has a dichotomous role in the regulation of cancer, increasing studies have shown the prosurvival role of autophagy in cancer progression and metastasis [28]. lncRNAs participate in the regulation of tumors and can be used as a molecular marker to predict the prognosis of patients with cancers [29]. Studies have shown that lncRNAs play a vital role in the development of ESCA [30–32]; however, there are no reports on autophagy-related lncRNA models that can predict the survival of patients with ESCA.

In this study, we constructed a coexpression network of lncRNAs and autophagy-related genes and used Cox regression analysis to identify four autophagy-related lncRNAs that might affect the prognosis of ESCA, specifically AC092718, FENDRR, LINC02381, and SEMA3B-AS1. We constructed an ESCA autophagy-related lncRNA risk assessment model and analyzed the correlation between the lncRNA model and the clinical characteristics and survival rate in patients with ESCA (Figure 8).

The article "Establishment and Analysis of a Prognostic Model of Autophagy-Related lncRNAs in ESCA" was published in 2022. Journal: Biomed Res Int.

AC092718.4 is a positive predictor of ovarian cancer and can play a role in cancer-related biological processes through a lncRNA–miRNA–mRNA regulatory network, such as cell cycle regulation, chromatin binding, modification, and remodeling the mTOR signaling pathway and the ovarian-specific *BRCA1*-related genome surveillance complex [33]. FENDRR, a lethal noncoding developmental regulatory RNA in the fetus, has been explored for its role in various cancers. In gastric cancer, FENDRR inhibits cell invasion and migration by downregulating fibronectin 1, and its low expression is associated with poor prognosis [34]. In breast cancer, FENDRR inhibits cell proliferation and is associated with a good prognosis [35]. In colorectal adenocarcinoma, the high FENDRR expression indicates a poor survival rate and promotes autophagy, apoptosis, and aging [36]. LINC02381 can be used as an oncogenic lncRNA and a tumor suppressor in cancer. It can aggravate the malignant phenotype and behavior of glioma cells by regulating the CBX5 expression. LINC02381 knockdown inhibits the malignant behavior of glioma cells and increases their proliferation [37]. In addition, LINC02381 is persistently expressed at low levels in breast cancer tissues, which might be related to immunity [38]. In gastric cancer tissues, the LINC02381 expression is downregulated, and its increased expression inhibits the activity of the Wnt pathway and cell cycle, increases cell apoptosis and caspase activity, and reduces the cell survival rate and proliferation rate of the human gastric cancer cell lines AGS and MKN45 [39]. SEMA3B-AS1 is a tumor suppressor lncRNA in cardia adenocarcinoma [40]. In hepatocellular carcinoma, the overexpression of SEMA3B-AS1 reduces hepatocellular carcinoma cell proliferation [41]. Additionally, SEMA3B-AS1 is significantly downregulated in ESCA, and its expression is related to TNM staging and lymph node metastasis. The SEMA3B-AS1 overexpression inhibits ESCA cell viability and invasiveness [42].

Our autophagy-related lncRNA signature could accurately predict the prognosis of patients with ESCA. This signature could be an independent indicator of ESCA, as revealed by univariate and multivariate Cox analyses. C-index and ROC curve analyses indicated that the model showed good discrimination and accuracy, suggesting that it might serve as a potential predictive method for patients with ESCA. GO analysis suggested that the selected lncRNAs were involved in the biological process of autophagosome assembly and autophagosome organization. Pathway enrichment analysis of downstream genes was also reported to be associated with autophagy and pathways in cancer. The results of functional enrichment analysis further confirmed that these prognostic autophagy-related lncRNAs play a role by regulating autophagy (Figure 8).

The article "Establishment and Analysis of a Prognostic Model of Autophagy-Related lncRNAs in ESCA" was published in 2022. Journal: Biomed Res Int.

This study had some limitations. First, the data used in this study were based on TCGA and HADb databases which are limited; therefore, the analysis results might be biased. Second, we did not verify the expression of these four lncRNAs in ESCA. We plan to prospectively collect patients and conduct follow-up to construct a test cohort to further validate the accuracy of the model in the next stage. Third, functional experiments have not been performed, and the potential molecular mechanism associated with the predictive effect of autophagy-related lncRNAs remains unclear.

In conclusion, the prognostic model established in this study provided an effective basis to reveal the function of lncRNAs related to autophagy in ESCA. We identified four autophagy-related lncRNAs that were significantly related to the prognosis of patients with ESCA and can be used to distinguish among patients with different risk statuses. Therefore, these four autophagy-related lncRNAs and their markers could serve as molecular biomarkers and therapeutic targets for patients with ESCA.

## 5. Conclusions

This study established an autophagy-related coexpression network of mRNAs and lncRNAs in ESCA and identified four genes with potential applications for the diagnostic and prognostic analysis of patients with ESCA. These data could provide new insights into the diagnosis and treatment of ESCA. We aim to investigate the specific mechanisms by which these genes regulate autophagy in future studies.

## Figures and Tables

**Figure 1:** (a) Differentially expressed lncRNAs in esophageal cancer. (b) Differentially expressed mRNAs in esophageal cancer. (c) Venn diagram showing the intersection of DEGs and HADb. (d) Venn diagram showing the intersection of DElncRNAs and ARlncRNAs (autophagy-related lncRNAs).

**Figure 2:** Survival analysis based on the four lncRNAs.

**Figure 3:** Multivariate Cox regression model analysis. (a) Overall survival curves for the four-gene combination in ESCA. (b) Risk scores: red indicates high risk, and green indicates low risk. (c) Survival diagram: red nodes indicate death, and green nodes indicate survival. (d) Heat map for the four-gene combination.

**Figure 4:** Coexpression network and Sankey diagram of the four prognostic autophagy-related lncRNAs. (a) Coexpression network of autophagy in Cytoscape; red indicates lncRNAs, and green indicates mRNAs. (b) Sankey diagram.

The article "Establishment and Analysis of a Prognostic Model of Autophagy-Related lncRNAs in ESCA" was published in 2022. Journal: Biomed Res Int.

**Figure 5:** Evaluation of prognostic models based on four autophagy-related lncRNAs. (a) Forest plots for (a) univariate and (b) multivariate Cox regression analyses in ESCA. (c) Nomogram of 3-year or 5-year overall survival based on the risk score, age, and TNM stage. (d) Receiver operating characteristic (ROC) curve analysis based on risk score and the clinicopathologic parameters.

**Figure 6:** PCA analysis based on the (a) expression profiles and (b) autophagy-related lncRNA prognostic signature.

**Figure 7:** Functional analysis. GO analysis using GSEA (a) and KEGG pathway (b) enrichment analysis.

**Figure 8:** Schematic diagram of the experimental design.

**Table 1:** Autophagy-related mRNAs (ARGmRNAs) and lncRNAs using correlation analysis.

ARGgene	lncRNA	cor	*P* value
BIRC5	MAFG-DT	0.46477	5.97*E*-10
ITPR1	AC007637.1	0.332063	1.79*E*-05
PRKAB1	AC007637.1	0.61085	9.73*E*-18
PRKAB1	AC091563.1	0.377207	8.80*E*-07
PRKAB1	AC004982.1	0.0318618	4.02*E*-05
ITPR1	FENDRR	0.790606	1.76*E*-35
GABARAPL1	FENDRR	0.308751	7.12*E*-05
ITPR1	AC037198.2	0.675193	1.23*E*-22
PINK1	AC092718.4	-0.33651	1.36*E*-05
PINK1	SNHG1	-0.35644	3.37*E*-06
BIRC5	SNHG1	0.341363	9.98*E*-06
PRKAB1	SEMA3B-AS1	0.312406	5.78*E*-05
ITPR1	ZNF710-AS1	0.413656	5.42*E*-08
PRKAB1	LINC02381	0.311697	6.02*E*-05

## Data Availability

The data that support the finding of this study are available from the corresponding upon the reasonable request.

## Abbreviations

ESCA: Esophageal cancer
lncRNA: Long noncoding RNA
mRNA: Messenger RNA
LC3: Light chain 3
HK2: Hexokinase 2
TCGA: The Cancer Genome Atlas
HADb: Human Autophagy Database
PCA: Principal component analysis
DEmRNA: Differently expressed mRNA
DElncRNA: Differentially expressed lncRNA
FC: Fold change
GSEA: Gene set enrichment analysis
GO: Gene Ontology
KEGG: Kyoto Encyclopedia of Genes and Genomes
HR: Hazard ratio
ROC: Receiver operating characteristic
AUC: Area under the curve
TNM: Tumor node metastasis.

## References

[1] Watanabe M., Otake R., Kozuki R. (2020). Recent progress in multidisciplinary treatment for patients with esophageal cancer. *Surgery Today*.

[2] Uhlenhopp D. J., Then E. O., Sunkara T., Gaduputi V. (2020). Epidemiology of esophageal cancer: update in global trends, etiology and risk factors. *Clinical Journal of Gastroenterology*.

[3] Papaefthymiou A., Christodoulidis G., Koffas A. (2021). Role of autophagy in gastric carcinogenesis. *World Journal of Gastrointestinal Oncology*.

[4] Colletti M., Ceglie D., Di Giannatale A., Nazio F. (2020). Autophagy and exosomes relationship in cancer: friends or foes?. *Frontiers in Cell and Development Biology*.

The article "Establishment and Analysis of a Prognostic Model of Autophagy-Related lncRNAs in ESCA" was published in 2022. Journal: Biomed Res Int.

[5] Liang J., Zhang L., Cheng W. (2021). Non-coding RNA-mediated autophagy in cancer: a protumor or antitumor factor?. *Biochimica Et Biophysica Acta. Reviews on Cancer*.

[6] Wu X., Zhou Z., Xu S. (2020). Extracellular vesicle packaged LMP1-activated fibroblasts promote tumor progression via autophagy and stroma-tumor metabolism coupling. *Cancer Letters*.

[7] Wu J., Gao F., Xu T. (2020). CLDN1 induces autophagy to promote proliferation and metastasis of esophageal squamous carcinoma through AMPK/STAT1/ULK1 signaling. *Journal of Cellular Physiology*.

[8] Amaravadi R., Kimmelman A. C., White E. (2016). Recent insights into the function of autophagy in cancer. *Genes & Development*.

[9] Kumar S., Sánchez-Álvarez M., Lolo F. N., Trionfetti F., Strippoli R., Cordani M. (2021). Autophagy and the lysosomal system in cancer. *Cell*.

[10] Saxena R., Klochkova A., Murray M. G. (2019). Roles for autophagy in esophageal carcinogenesis: implications for improving patient outcomes. *Cancers*.

[11] Camacho C. V., Choudhari R., Gadad S. S. (2018). Long noncoding RNAs and cancer, an overview. *Steroids*.

[12] Ulitsky I., Bartel D. P. (2013). lincRNAs: genomics, evolution, and mechanisms. *Cell*.

[13] Yang C., Chen K. (2022). Long non-coding RNA in esophageal cancer: a review of research progress. *Pathology Oncology Research*.

[14] Chen M. J., Deng J., Chen C., Hu W., Yuan Y. C., Xia Z. K. (2019). LncRNA H19 promotes epithelial mesenchymal transition and metastasis of esophageal cancer via STAT3/EZH2 axis. *The International Journal of Biochemistry & Cell Biology*.

[15] Ramli S., Sim M. S., Guad R. M. (2021). Long noncoding RNA UCA1 in gastrointestinal cancers: molecular regulatory roles and patterns, mechanisms, and interactions. *Journal of Oncology*.

[16] Liu H. E., Shi H. H., Luo X. J. (2020). Upregulated long noncoding RNA UCA1 enhances Warburg effect via miR-203/HK2 axis in esophagal cancer. *Journal of Oncology*.

[17] Zhang J., Hu S. L., Qiao C. H. (2018). LncRNA-NEF inhibits proliferation, migration and invasion of esophageal squamous-cell carcinoma cells by inactivating wnt/*β*-catenin pathway. *European Review for Medical and Pharmacological Sciences*.

[18] Yao J., Zhang H., Li H., Qian R., Liu P., Huang J. (2020). P53-regulated lncRNA uc061hsf.1 inhibits cell proliferation and metastasis in human esophageal squamous cell cancer. *IUBMB Life*.

[19] Chen D., Wang M., Xu Y. (2021). A novel autophagy-related lncRNA prognostic signature associated with immune microenvironment and survival outcomes of gastric cancer patients. *International Journal of General Medicine*.

[20] Frankel L. B., Lubas M., Lund A. H. (2017). Emerging connections between RNA and autophagy. *Autophagy*.

The article "Establishment and Analysis of a Prognostic Model of Autophagy-Related lncRNAs in ESCA" was published in 2022. Journal: Biomed Res Int.

[21] Sun T. (2018). Long noncoding RNAs act as regulators of autophagy in cancer. *Pharmacological Research*.

[22] Sheng S. R., Wu J. S., Tang Y. L., Liang X. H. (2017). Long noncoding RNAs: emerging regulators of tumor angiogenesis. *Future Oncology*.

[23] Kondo A., Nonaka A., Shimamura T. (2017). Long noncoding RNA JHDM1D-AS1 promotes tumor growth by regulating angiogenesis in response to nutrient starvation. *Molecular and Cellular Biology*.

[24] Wang M., Gu J., Zhang X., Yang J., Zhang X., Fang X. (2021). Long non-coding RNA DANCR in cancer: roles, mechanisms, and implications. *Frontiers in Cell and Development Biology*.

[25] Bolger J. C., Donohoe C. L., Lowery M., Reynolds J. V. (2021). Advances in the curative management of oesophageal cancer. *British Journal of Cancer*.

[26] Nagaki Y., Motoyama S., Yamaguchi T. (2020). m6A demethylase ALKBH5 promotes proliferation of esophageal squamous cell carcinoma associated with poor prognosis. *Genes to Cells*.

[27] Ganzleben I., Neurath M. F., Becker C. (2021). Autophagy in cancer therapy—molecular mechanisms and current clinical advances. *Cancers*.

[28] Das C. K., Banerjee I., Mandal M. (2020). Pro-survival autophagy: an emerging candidate of tumor progression through maintaining hallmarks of cancer. *Seminars in Cancer Biology*.

[29] Jin K. T., Lu Z. B., Lv J. Q., Zhang J. G. (2020). The role of long non-coding RNAs in mediating chemoresistance by modulating autophagy in cancer. *RNA Biology*.

[30] Zhang Y., Li R., Ding X., He M., Zhang R. (2022). Long noncoding RNA SNHG6 promotes oesophageal squamous cell carcinoma by downregulating the miR-101-3p/EZH2 pathway. *Journal of Biochemical and Molecular Toxicology*.

[31] Shen S., Liang J., Liang X. (2022). SNHG17, as an EMT-related lncRNA, promotes the expression of c-Myc by binding to c-Jun in esophageal squamous cell carcinoma. *Cancer Science*.

[32] Hu R., Bi R., Jiang L., Yang X., Zhong Y., Xie X. (2021). LncRNA TUSC8 suppresses the proliferation and migration of esophageal cancer cells by downregulation of VEGFA. *Journal of Cancer*.

[33] Lin N., Lin J. Z., Tanaka Y., Sun P., Zhou X. (2021). Identification and validation of a five-lncRNA signature for predicting survival with targeted drug candidates in ovarian cancer. *Bioengineered*.

[34] Xu T. P., Huang M. D., Xia R. (2014). Decreased expression of the long non-coding RNA FENDRR is associated with poor prognosis in gastric cancer and FENDRR regulates gastric cancer cell metastasis by affecting fibronectin1 expression. *Journal of Hematology & Oncology*.

[35] Li Y., Zhang W., Liu P. (2018). Long non-coding RNA FENDRR inhibits cell proliferation and is associated with good prognosis in breast cancer. *Oncotargets and Therapy*.

The article "Establishment and Analysis of a Prognostic Model of Autophagy-Related lncRNAs in ESCA" was published in 2022. Journal: Biomed Res Int.

[36] Yang F., Sun S., Yang F. (2021). Prognostic and predicted significance of FENDRR in colon and Rectum adenocarcinoma. *Frontiers in Oncology*.

[37] Sun Y., Wang X., Bu X. (2021). LINC02381 contributes to cell proliferation and hinders cell apoptosis in glioma by transcriptionally enhancing CBX5. *Brain Research Bulletin*.

[38] Ghafouri-Fard S., Asadi M., Sohrabi B. (2021). Down-regulation of a panel of immune-related lncRNAs in breast cancer. *Pathology, Research and Practice*.

[39] Jafarzadeh M., Soltani B. M. (2020). Long noncoding RNA LOC400043 (LINC02381) inhibits gastric cancer progression through regulating Wnt signaling pathway. *Frontiers in Oncology*.

[40] Guo W., Liang X., Liu L. (2019). MiR-6872 host gene SEMA3B and its antisense lncRNA SEMA3B-AS1 function synergistically to suppress gastric cardia adenocarcinoma progression. *Gastric Cancer*.

[41] Zhong Y., Li Y., Song T., Zhang D. (2019). MiR-718 mediates the indirect interaction between lncRNA SEMA3B-AS1 and PTEN to regulate the proliferation of hepatocellular carcinoma cells. *Physiological Genomics*.

[42] Dong Z., Liang X., Wu X. (2019). Promoter hypermethylation-mediated downregulation of tumor suppressor gene SEMA3B and lncRNA SEMA3B-AS1 correlates with progression and prognosis of esophageal squamous cell carcinoma. *Clinical & Experimental Metastasis*.

